RETRACTED

# Prophylactic Use of Antibiotics for Postsurgical Infection in c-TACE and DEB-TACE High-Risk Patients: A Case-Control Study

**DOI:** 10.1155/2022/6203817

**Published:** 2022-04-11

**Authors:** Baojian Li

**Affiliations:** Department of Pharmacy, Heping Hospital Affiliated to Changzhi Medical College, Changzhi 046000, Shanxi, China

## Abstract

**Objectives:**

According to recent reports, prophylactic use of antibiotics is not always required in conventional transarterial chemoembolization (c-TACE). However, clinical evidence of prophylactic antibiotics in drug-eluting beads transarterial chemoembolization (DEB-TACE) to prevent postsurgical infection is limited. This study is aimed to evaluate the correlation between the preoperative prophylactic application of antibiotics and postoperative infection in c-TACE or DEB-TACE, especially in a population with a high risk for postsurgical infection.

**Methods:**

In this retrospective study, TACE patients diagnosed with hepatic carcinoma (between January 2019 and May 2021) were examined. The case group was given 1.5 g cefuroxime sodium 0.5–1 hour before TACE, while there was no intervention in the control group. The outcomes analyzed were leukocyte count >9.5 × 10^9^/L on the second day after the operation and the diagnosis of infection within one month after the operation. We applied univariate, multivariate logistic regression, trend analysis, and subgroup analysis to find potential risk factors and the necessity of prophylactic antibiotics.

**Results:**

Among 142 eligible cases, 72 received antibiotics while 70 were kept as control, 113 cases were treated with c-TACE, and 29 were treated with DEB-TACE. Multivariate analysis showed that the increase in white blood cell count after the operation was related to diabetes (OR 5.112, 95% CI 1.229–21.264, *p* = 0.025). The occurrence of postoperative infection was negatively correlated with preoperative albumin value (＜25 g/L) (OR 153.118, 95% CI 1.631–14372.331, *p* = 0.030). Trend analysis showed that the risk of postoperative infection increased with a decrease in serum albumin level (*P* < 0.05). Subgroup analysis showed that there were no significant differences in the incidence of increased leukocyte count and postoperative infection between the prophylactic and nonprophylactic treatment groups, in the case of diabetes, preoperative albumin levels, and operation mode (*P* > 0.1).

**Conclusions:**

Prophylactic antibiotic treatment before the c-TACE or DEB-TACE had no significant correlation with postoperative leukocyte increase and postoperative infection. Diabetes history and serum albumin levels were the prominent risk factors associated with an increase in postoperative leukocyte count and postoperative infection. Future large-scale studies and randomized-controlled trials are required to confirm and validate this association.

RETRACTED

## 1. Introduction

Liver cancer especially hepatocellular carcinoma (HCC) is among the top five most common cancers. The treatment of HCC includes surgery, liver transplantation, and radiofrequency ablation with good survival benefits. However, most HCC patients having vascular involvement or multiple lesions cannot be treated with such treatment strategies [1]. Transarterial chemoembolization (TACE) is the currently known standard of care treatment of HCC in intermediate-stage patients and the most widely used nonsurgical method for the treatment of liver cancer [2]. TACE is divided into conventional TACE (c-TACE) and drug-elating beads TACE (DEB-TACE) [3, 4]. In c-TACE, a mixture of anticancer agents (e.g., cisplatin and doxorubicin) in the lipid-based formulation is administered to liver cancer patients for the treatment of intermediate-stage cancer. The foundation of this treatment is based on the recommendations of the systemic review of randomized-controlled trials (RCTs) [5]. On the other hand, in drug-eluting beads TACE, the anticancer drugs are delivered to the target site in a delivery system which combines local embolization of vasculature and release of the anticancer drug in nearby tissues [6, 7]. This procedure is specifically applied in patients with hypervascular tumors for the treatment of cancer. The administration procedure of DEB-TACE is nearly similar to c-TACE, and both are minimally invasive procedures usually carried out by radiologists [8]. The beads employed in DEB-TACE are mainly biocompatible polymers-based hydrogels including polyvinyl alcohol (PVA)-based hydrogels which are sulphonated for binding of anticancer drugs [9]. The anticancer agents are delivered to the target site upon occlusion of the beads in the vasculature, which embolizes them, and subsequently, the drug is released in the target site [10]. It is currently unclear whether DEB-TACE or c-TACE should be used for a specific patient in the absence of randomized-controlled trials. However, DEB-TACE has a safer profile than c-TACE, with fewer common side effects [3, 4, 11, 12]. Therefore, the application of DEB-TACE is becoming more and more extensive.

TACE procedures have been regarded as minimally invasive with a good curative profile and strong repeatability; thus, it is mostly used in the nonsurgical treatment of HCC. However, the chance of occurrence of infection is always there, which results will not only prolong the hospital stay and expenses but also will affect the efficacy of treatment [13]. Moreover, the majority of the TACE-treated patients are middle-aged, or they are in the advanced stage of cancer where the immune system is less active, coupled with damage to nearby tissues caused by operation and the anticancer drugs' immune function inhibition leading to postoperative infection [14, 15].

RETRACTED

It is uncertain whether the use of antibiotics as prophylaxis before TACE is beneficial or not in the prevention of postoperative infection. The guidelines for the use of antibiotics in the China interventional radiology department believe that prophylactic use of antibiotics is generally not necessary. But if the patient has a poor physique, low immunity, and a history of biliary surgery, antibiotics can be used for prevention before the operation. The guiding principles for the clinical application of antibiotics in China suggest that antibiotics should be used to prevent infection before TACE [16]. According to Yoshihara et al., prophylactic antibiotic treatment in patients having TACE was linked to a lower risk of liver abscess necessitating surgical intervention [17]. However, recent findings show that prophylactic antibiotic medication is not always required in the TACE process for HCC patients [15, 18]. Moreover, serum albumin level, white blood cell count, length of stay, skin or mucosal ulcer, invasive operation, application of broad-spectrum antibiotics, and diabetes mellitus were independent risk factors for nosocomial infection after TACE in patients with primary liver cancer [15, 19].

The above studies on the preventive application of antibiotics refer to c-TACE or are not explicitly stated. Whether DEB-TACE needs to prevent the use of antibiotics before the operation has not been recommended by guidelines or relevant studies, and whether there are the same risk factors related to the prevention of the use of antibiotics with c-TACE has not been reported. It has been reported that postoperative infections such as a liver abscess occurred after DEB-TACE [20–22].

The abuse and unnecessary use of antibiotics has become a worldwide problem. It not only increases the occurrence and cost of adverse drug reactions but also is considered to be one of the main reasons for the emergence of more and more biological drug-resistant strains [23]. Optimizing the antibiotic prevention strategy in the TACE treatment of hepatocellular carcinoma is necessary and urgent not only for patients with hepatocellular carcinoma but also for the whole population. The value of routine prophylaxis merits justification [24].

This study aimed to explore the relationship between the use of antibiotics and postoperative infection not only in c-TACE but also in DEB-TACE, using logistic regression and trend analysis. Subgroup analysis was also conducted to study the interaction and confounding factors between high-risk factors and preventive drug use outcomes.

RETRACTED

## 2. Methods

### 2.1. Ethical Considerations

The reports were in accordance with the Strengthening the Reporting of Observational Studies in Epidemiology (STROBE) guideline. The approval for the current retrospective study was provided by the Ethics Committee of the Heping Hospital Affiliated to Medical College, Changzhi, China. Informed consent was not required because of the retrospective nature of the study and the anonymity of the collected data.

### 2.2. Data Source and Patients

Between January 2019 and May 2021, the data of patients with primary liver malignancies, hepatocellular carcinoma (HCC), intrahepatic cholangiocarcinoma (ICC) [25, 26], and metastatic liver malignancies treated with TACE at Heping Hospital Affiliated with Changzhi Medical College were retrospectively analyzed. The laboratory examination data were obtained from the clinical laboratory of the hospital, and other results were accessed from the medical record system of the hospital.

### 2.3. Inclusion and Exclusion Criteria

The control and case inclusion criteria was based on the indications and contraindications of TACE treatment following the guidelines for diagnosis and treatment of primary liver cancer in China (Edition 2019) [25]. The cases of c-TACE were given iodized oil-based chemotherapeutic drug emulsions, supplemented with granular embolic agents. Granular embolic agents included gelatin sponge particles, blank microspheres, and polyvinyl alcohol particles. The DEB-TACE cases were given a therapeutic scheme of embolization with CalliSpheres drug-loaded microspheres (100–300 *μ*m) preloaded with chemotherapeutic drugs. The case group was given 1.5 g cefuroxime sodium for injection only once 0.5–1 hour before TACE, while the control group had no preventive medication before TACE. Patients with incomplete or missing laboratory tests data were excluded from the analyses.

### 2.4. Outcomes

The outcomes assessed in this study were as follows:

1. Increase in leukocyte count (>9.5 × 10^9^/L) on the second day after the operation
2. The diagnosis of infection within one month after the operation was based on the diagnostic criteria of hospital infection and diagnostic criteria of nosocomial infection (China, 2001) [27].

### 2.5. Statistical Analysis

All statistical analyses were conducted using SPSS (V.26.0; IBM). A univariate analysis was employed for the comparison of variations in patients' baseline characteristics between the preventive medication group and the nonpreventive medication group. The Student's *t*-test was employed to evaluate if the obtained data had a homogeneous variance and a normal distribution. For nonhomogeneous variance, the comparisons were made using a one-way analysis of variance (ANOVA). In order to compare categorical variables, Fisher's exact test or Pearson's 2 test was used as applicable.

RETRACTED

Then, univariate analysis was used to compare the clinical data which is between the WBC≤9.5×109/L group and the WBC＞9.5×109/L group and between the nonpostoperative infection group and the postoperative infection group to find associated variables, respectively. The univariate analysis included chi-square tests for categorical variables and *t*-tests for continuous variables. Significant variables (*P* < 0.01) in univariate analysis and covariates considered clinically influential were then analyzed by multivariate stepwise logistic regression (forward stepwise logistic regression) to identify significant variables. We applied univariate and multivariate logistic regression models to estimate odds ratios (ORs) with 95% confidence intervals (CIs) for significant variables for finding potential risk factors in WBC＞9.5×109/L group or postoperative infection group. In addition, dummy variables are set for grade data to test its trend.

Finally, Cochran's and mantel Haenszel tests were used for subgroup analysis of high-risk factors and surgical methods to determine whether there were important variables affecting the outcome of preoperative preventive drug treatment. *P* value less than 0.05 was considered statistically significant.

## 3. Results

A total of 103 patients underwent 145 TACE. Three of these patients were lacking blood sample data and were excluded from data analysis (Figure 1). The remaining 102 patients who underwent 142 procedures were included in the analysis. All the patients were diagnosed with primary liver cancer, according to the criteria mentioned earlier. The baseline characteristics of patients are listed in Table 1, and no significant difference was found between the preventive medication (*n* = 72) group and nonpreventive medication (*n* = 70) group (*p* > 0.05).

### 3.1. Univariate Analysis of Outcomes

There were 28 cases with postoperative leukocyte count >9.5 × 10^9^/L. Patients with diabetes history, age ranges, or preoperative albumin value (≥25 g/L, ＜40 g/L) showed significant associations with postoperative leukocyte count >9.5 ×109/L (*P* < 0.1). There were 14 cases of postoperative infection. Patients with gallstone, number of TACE, or preoperative albumin value (＜25 g/L) showed significant associations with postoperative infection (*P* < 0.1). There was no significant correlation between preoperative prophylactic medication or operation mode and postoperative leukocyte count or postoperative infection (*P* > 0.1) as shown in Table 2.

RETRACTED

### 3.2. Multivariate Analysis of Outcomes

The increase in white blood cell count after the operation was related to diabetes history (OR 5.112, 95% CI 1.229–21.264, *p* = 0.025), which was unrelated to the age of the patients (*P* > 0.05). The occurrence of postoperative infection was related to the preoperative albumin value (＜25 g/L) (OR 153.118, 95% CI1.631–14372.331, *p* = 0.030), and there was no significant correlation with gallstone (OR 3.626, 95% CI 0.843–15.597, *p* = 0.084) and number of TACE (OR 0.394, 95% CI 0.154–1.005, *p* = 0.051) as shown in Table 2.

### 3.3. Trend Analysis of Outcomes

The trend analysis of outcomes showed that the risk of increased leukocyte count was not related to the age of the patients with no statistically significant trend (trend *P* > 0.05). The risk of postoperative infection increased with a decrease in albumin level, which was statistically significant with or without adjustment variables (*P* < 0.05) as shown in Table 2.

### 3.4. Subgroup Analysis of Outcomes

Multivariate analysis revealed that the potential confounding factors were diabetes history and preoperative albumin levels. A surgical method that is considered clinically influential also needs hierarchical analysis. Two out of four patients with a history of diabetes with no prophylactic medication showed white blood cells' count of >9.5 × 10^9^/L as shown in Table 3. On the other hand, 3 out of 9 patients with diabetic history and prophylactic medication showed an increase in leukocyte count. The effect of albumin level and different surgical methods on the preoperative infection was analyzed, and the results are shown in Table 4. It is evident from the table that the maximum number of patients with albumin levels below 25 g/L experienced postoperative infection. The surgical method applied had no effect on the postoperative infection. The effect of diabetes mellitus, preoperative albumin levels, and operation mode on the increase in WBC count or postoperative infection was also assessed. The results are shown in Table 5 which indicates that there was no significant difference in postoperative infection or increase in WBC counts between the prophylactic and nonpreventive treatment groups, diabetes mellitus, preoperative albumin levels, or operation mode (*P* > 0.1).

## 4. Discussion

This study retrospectively analyzed the need for preoperative prophylactic use of antibiotics in patients who underwent c-TACE and DEB-TACE. The results showed that there were no significant differences in the incidence of increased leukocytes count and postoperative infection with both applied surgical methods. However, the history of diabetes and preoperative serum albumin level were risk found factors for postoperative leukocyte elevation and postoperative infection. However, these factors cannot alter the effect of prophylactic use of antibiotics before c-TACE or DEB-TACE on postoperative leukocyte elevation and postoperative infection.

RETRACTED

The need for prophylactic use of antibiotics before c-TACE is consistent with the previous research results [18, 28, 29]. The risk factors for postoperative infection, such as diabetes history [19] and preoperative serum albumin level [15], are also consistent with previous studies. Some studies have shown that the risk of postoperative infection increases with the increase of age [30], but our results show there was no significant difference between age and postoperative leukocyte count or postoperative infection. This may be related to fewer positive cases of postoperative infection, and more cases are needed to prove it. Some studies have shown that biliary surgery is a risk factor for postoperative infection [31]. TACE can be performed without antibiotics in patients with intact biliary anatomy [24]. Our study did not find that biliary surgery is related to postoperative infection, which may be related to fewer cases of biliary surgery. Our study found that cholecystolithiasis is an independent risk factor for postoperative infection, but it cannot change the effect of preoperative medication on postoperative infection.

We clearly distinguished between therapeutic and prophylactic antibiotics and control the dose and timing of prophylactic antibiotics. The cases we included did not undergo pathological typing screening, which is applicable to all patients with liver malignant tumors treated with TACE. It can also be used as a reference for the preoperative preventive medication of DEB-TACE (CalliSpheres drug-loaded microspheres 100–300 um). This research was carried out at Changzhi, China, where the minimum inhibitory concentration of cefuroxime sodium for most *Escherichia coli* (E Coli), *Staphylococcus aureus*, and *Klebsiella* pneumonia is low. Keeping the above-mentioned points in mind, the findings of our study may not be applicable to places where resistant bacteria are prevalent in high or low numbers. More instances should be included in the future to better understand the need for antibiotics to be used as a prophylactic measure.

## 5. Limitations of the Study

In this study, fewer cases, especially very less cases with positive outcomes, were included. To generalize the results of this study, more case studies and randomized-controlled trials are needed.

RETRACTED

In addition, this study was carried out in an area where the minimum inhibitory concentration of the antibiotic (cefuroxime sodium) is very low against E. Coli, K. pneumonia, and *S. aureus*. Therefore, the results of this study may not be applicable to places where resistant bacterial strains are prevalent. Moreover, in this study, the cases of DEB-TACE were CalliSpheres 100–300 *μ*m microsphere preloaded with chemotherapeutic drugs. According to Prajapati et al., the use of 100–300 m sized particles is associated with a much-improved survival rate and fewer problems when compared to the use of 300–500 and 500–700 m sized DEB [32]. Therefore, it cannot represent other drug-loaded microspheres precisely. Thus, it is suggested to conduct and include cases of DEB size 300–500 and 500–700 m in other large studies to get conclusive and evidence-based results.

## 6. Conclusion

This study was aimed to analyze the effect of prophylactic use of antibiotics on the postoperative leukocytes count in a population with high risk factors for postsurgical infection undergoing c-TACE and DEB-TACE. Results of this study showed that prophylactic antibiotic treatment before the c-TACE or DEB-TACE had no significant correlation with the postoperative increase in leukocyte count and postoperative infection. Diabetes history and serum albumin levels were the prominent risk factors associated with an increase in postoperative leukocyte count and postoperative infection. If a patient has a history of diabetes during the c-TACE treatment or a serum albumin level <25 g/L during DEB-TACE treatment, antibiotics are recommended to prevent postoperative infection. Future large-scale studies and randomized-controlled trials are required to confirm and validate this association.

## Figures and Tables

**Figure 1:** Allocation of subjects to case and control groups.

**Table 1:** Population and baseline characteristics.

Baseline characteristics	Preventive medication group	Nonpreventive medication group	*P*-value
Numbers	72	70	
Age (years)	61.43 ± 9.805	60.19 ± 8.742	0.426
Sex (male/female)	54/18	59/11	0.170
Diabetes history (yes/no)	9/63	4/66	0.161
History of biliary surgery (yes/no)	6/66	8/62	0.536
Gallstone (yes/no)	12/60	8/62	0.370
Operation mode (c-tace/deb-tace)	60/12	53/17	0.260
Number of TACE (n)			0.691
First time	33	29	
Second time	19	22	
Third time	10	6	
Fourth time	2	6	
Fifth time	4	3	
Sixth time	1	1	
Seventh time	1	1	
Ninth time	1	1	
Tenth time	1	0	
Eleventh time	0	1	
Preoperative albumin value (g/L)	34.654 ± 5.0938	34.817 ± 4.4169	0.839
Preoperative leukocyte count (10^9^/L)	5.193 ± 2.2486	5.268 ± 1.8230	0.831

RETRACTED

**Table 2:** Univariate, multivariate, and trend analysis of outcomes.

Variables	Postoperative leukocyte count >9.5 × 10^9^/L group (*n* = 28)				Postoperative infection group (*n* = 14)			
	Univariate analysis		Multivariate analysis		Univariate analysis		Multivariate analysis	
	*p* value	Odds ratio (95% CI)	*p* value	Odds ratio (95% CI)	*p* value	Odds ratio(95% CI)	*p* value	Odds ratio(95% CI)
Age (years)	0.093^*∗*^	0.705(0.470–1.060)	0.152^*∗*^	0.720(0.460–1.128)				
≤ 39	0.050	14.677(0.999–215.310)	0.073	16.087(0.776–333.645)	0.176	4.444(0.512–38.611)		
40–49	0.139	6.000(0.557–64.576)	0.126	7.462(0.568–98.016)	0.581	0.513(0.048–5.477)		
50–59	0.094	6.286(0.730–54.099)	0.073	8.022(0.825–78.002)	0.823	0.833(0.169–4.118)		
60–69	0.088	6.160(0.762–49.793)	0.061	8.257(0.909–75.019)	0.314	0.444(0.092–2.518)		
70+	Reference		Reference		Reference		Reference	
Sex (male/female)	0.883	0.927(0.337–2.549)			0.223	3.640(0.456–29.039)		
Diabetes history (yes/no)	0.085	2.880(0.863–9.610)	0.025	5.112(1.229–21.264)	0.488	1.773(0.351–8.954)		
History of biliary surgery (yes/no)	0.593	0.654(0.138–3.104)			0.999	0.000(0.000–0.000)		
Gallstone (yes/no)	0.973	1.021(0.313–3.332)			0.003	6.107(1.848–20.179)	0.084	3.626(0.843–15.597)
Operation mode (c-tace/deb-tace)	0.504	1.394(0.526–3.691)			0.922	1.070(0.278–4.116)		
Number of TACE (n)	0.919	0.988(0.788–1.240)			0.075	0.515(0.248–1.068)	0.051	0.394(0.154–1.005)
Preoperative albumin value (g/L)	0.270^*∗*^	0.566(0.206–1.556)	0.289^∗^	0.5610.192–1.633)	0.011^*∗*^	11.097(1.738–70.873)	0.046 ^*∗*^	8.824(1.041–74.773)
≥40 g/L	Reference				Reference		Reference	
≥25 g/L,＜40 g/L	0.037	0.326(0.114–0.934)	0.082	0.364(0.117–1.136)	0.642	1.651(0.199–13.693)	0.455	2.332(0.253–21.472)
＜25 g/L	0.626	1.714(0.196–15.019)	0.821	1.335(0.110–16.147)	0.010	54.000(2.611–11116.898)	0.030	153.118(1.631–14372.331)
Preoperative preventive medication (yes/no)	0.614	0.808(0.353–1.850)			0.290	1.857(0.590–5.847)		

^*∗*^  = *p* for trend.

**Table 3:** Number of subgroup cases in diabetes and in operation mode.

Diabetes history/operation mode	Whether preventive medication	Postoperative leukocyte count normal	Postoperative leukocyte count >9.5 ×109/L	Total
Nondiabetes history	N	53	13	66
	Y	53	10	63
	Total	106	23	129
Diabetes history	N	2	2	4
	Y	6	3	9
	Total	8	5	13
Total	N	55	15	70
	Y	59	13	72
	Total	114	28	142
c-TACE	N	42	11	53
	Y	50	10	60
	Total	92	21	113
DEB⁃TACE	N	13	4	17
	Y	9	3	12
	Total	22	7	29
Total	N	55	15	70
	Y	59	13	72
	Total	114	28	142

**Table 4:** Number of subgroup cases in preoperative albumin value and in operation mode.

Preoperative albumin value (g/L)/operation mode	Whether preventive medication	Non postoperative infection	Postoperative infection	Total
≥40	N	8	0	8
	Y	10	1	11
	Total	18	1	19
≥25-＜40	N	56	4	60
	Y	53	6	59
	Total	109	10	119
＜25	N	1	1	2
	Y	0	2	2
	Total	1	3	4
Total	N	65	5	70
	Y	63	9	72
	Total	128	14	142
c-TACE	N	49	4	53
	Y	53	7	60
	Total	102	11	113
DEB⁃TACE	N	16	1	17
	Y	10	2	12
	Total	26	3	29
Total	N	65	5	70
	Y	63	9	72
	Total	128	14	142

RETRACTED

**Table 5:** Subgroup analysis of preventive medication group and nonpreventive medication group.

Outcome event	High risk factors	Cochran's		Mantel-Haenszel			Mantel-Haenszel common odds ratio	
		Chi-squared	Asymptotic significance (2-sided)	Chi-squared	Asymptotic significance (2-sided)	Odds ratio (95% CI)	Odds ratio (95% CI)	Asymptotic significance (2-sided)
Postoperative leukocyte count >9.5 × 10^9^/L	Diabetes history (yes/no)	0.534	0.465	0.261	0.61	0.808 (0.353–1.850)	0.730 (0.312–1.706)	0.467
	Operation mode (c-tace/deb-tace)	0.198	0.657	0.053	0.818	0.808 (0.353–1.850)	0.829 (0.361–1.903)	0.658
Postoperative infection	Preoperative albumin value (g/L)	1.256	0.262	0.649	0.420	1.857 (0.590–5.847)	1.886 (0.593–6.000)	0.282
	Operation mode (c-tace/deb-tace)	1.177	0.278	0.634	0.426	1.857 (0.590–5.847)	1.864 (0.593–5.857)	0.287

## Data Availability

The data will be provided upon request to the authors.

## References

[1] Chan W.-H., Huang S.-F., Lee C.-W. (2019). Incorporation of biochemical factors for survival analysis of transarterial chemoembolization in patients with hepatocellular carcinoma: a retrospective cohort study. *Journal of International Medical Research*.

[2] Sieghart W., Hucke F., Peck-Radosavljevic M. (2015). Transarterial chemoembolization: modalities, indication, and patient selection. *Journal of Hepatology*.

[3] Zou J. H., Zhang L., Ren Z. G., Ye S. L. (2016). Efficacy and safety of cTACEversusDEB-TACE in patients with hepatocellular carcinoma: a meta-analysis. *Journal of Digestive Diseases*.

[4] Melchiorre F., Patella F., Pescatori L. (2018). DEB-TACE: a standard review. *Future Oncology*.

[5] Llovet J., Bruix J. (2003). Systematic review of randomized trials for unresectable hepatocellular carcinoma: chemoembolization improves survival. *Hepatology*.

[6] Lewis A. L., Taylor R. R., Hall B., Gonzalez M. V., Willis S. L., Stratford P. W. (2006). Pharmacokinetic and safety study of doxorubicin-eluting beads in a porcine model of hepatic arterial embolization. *Journal of Vascular and Interventional Radiology*.

[7] Lewis A. L., Gonzalez M. V., Lloyd A. W. (2006). DC bead: in vitro characterization of a drug-delivery device for transarterial chemoembolization. *Journal of Vascular and Interventional Radiology*.

[8] Shi Q., Chen D., Zhou C. (2020). Drug-eluting beads versus lipiodol transarterial chemoembolization for the treatment of hypovascular hepatocellular carcinoma: a single-center retrospective study. *Cancer Management and Research*.

RETRACTED

[9] Tang Y., Taylor R., Gonzalez M., Lewis A., Stratford P. (2006). Evaluation of irinotecan drug-eluting beads: a new drug–device combination product for the chemoembolization of hepatic metastases. *Journal of Controlled Release*.

[10] Liu K.-C., lv W.-F., Lu D. (2021). Initial experience of drug-eluting bead-transcatheter arterial chemoembolization after lipiodol-based transcatheter arterial chemoembolization failure for patients with advanced hepatocellular carcinoma. *Cancer Management and Research*.

[11] Facciorusso A. (2018). Drug-eluting beads transarterial chemoembolization for hepatocellular carcinoma: current state of the art. *World Journal of Gastroenterology*.

[12] Fohlen A., Tasu J. P., Kobeiter H., Bartoli J. M., Pelage J. P., Guiu B. (2018). Transarterial chemoembolization (TACE) in the management of hepatocellular carcinoma: results of a French national survey on current practices. *Diagnostic and interventional imaging*.

[13] Kang S. J., Kim U. J., Kim S. E. (2018). Predictive value of procalcitonin for bacterial infection after transarterial chemoembolization or radiofrequency ablation for hepatocellular carcinoma. *Disease Markers*.

[14] Dutta R., Mahato R. I. (2017). Recent advances in hepatocellular carcinoma therapy. *Pharmacology & Therapeutics*.

[15] Shi Z., Yang W., Tang H., Li X. (2021). Risk factors of infection after transarterial chemoembolization for hepatocellular carcinoma: a protocol for systematic review and meta-analysis. *Medicine*.

[16] Association C. M., Association P. P. A. C. O. C. H., Association H. P. A. C. O. C. P. (2005). Guiding principles for clinical application of antibiotics. *Adver Drug React J*.

[17] Yoshihara S., Yamana H., Akahane M. (2021). Association between prophylactic antibiotic use for transarterial chemoembolization and occurrence of liver abscess: a retrospective cohort study. *Clinical microbiology and infection: The Official Publication of the European Society of Clinical Microbiology and Infectious Diseases*.

[18] Plentz R. R., Lankisch T. O., Bastürk M. (2005). Prospective analysis of German patients with hepatocellular carcinoma undergoing transcatheter arterial chemoembolization with or without prophylactic antibiotic therapy. *Journal of Gastroenterology and Hepatology*.

[19] Nouri Y. M., Kim J. H., Yoon H.-K., Ko H.-K., Shin J. H., Gwon D. I. (2019). Update on transarterial chemoembolization with drug-eluting microspheres for hepatocellular carcinoma. *Korean Journal of Radiology*.

[20] Toro A., Bertino G., Arcerito M. C. (2015). A lethal complication after transarterial chemoembolization with drug-eluting beads for hepatocellular carcinoma. *Case Reports in Surgery*.

RETRACTED

[21] Ye T., Zhu P., Liu Z., Ren Q., Zheng C., Xia X. (2022). Liver abscess after drug-eluting bead chemoembolization in patients with metastatic hepatic tumors. *British Journal of Radiology*.

[22] Woo S., Chung J. W., Hur S. (2013). Liver abscess after transarterial chemoembolization in patients with bilioenteric anastomosis: frequency and risk factors. *American Journal of Roentgenology*.

[23] Nepal G., Bhatta S. (2018). Self-medication with antibiotics in WHO southeast asian region: a systematic review. *Cureus*.

[24] Watchmaker J. M., Lipnik A. J., Fritsche M. R. (2018). Are prophylactic antibiotics necessary prior to transarterial chemoembolization for hepatocellular carcinoma in patients with native biliary anatomy?. *Journal of Surgical Oncology*.

[25] Zhou J., Sun H., Wang Z. (2020). Guidelines for the diagnosis and treatment of hepatocellular carcinoma (2019 Edition). *Liver Cancer*.

[26] of Interventionalists C. C., Association C. M. D. (2019). Chinese Clinical Practice Guidelines for transarterial chemoembolization of hepatocellular carcinoma. *Zhonghua gan zang bing za zhi= Zhonghua ganzangbing zazhi= Chinese journal of hepatology*.

[27] China M. O. H. O. T. P. S. R. O. (2001). Diagnostic criteria for nosocomial infections. *Chinese Medical Journal*.

[28] Ebisutani C., Sato S., Nishi K., Inoue H., Yoshie T., Kinoshita Y. (2010). Antibiotic prophylaxis in transcatheter treatment of hepatocellular carcinoma: an open randomized prospective study of oral versus intravenous administration. *Internal Medicine*.

[29] Chen J., Wu G. (2018). Retrospective analysis of Chinese patients with hepatocellular carcinoma (HCC) undergoing transcatheter arterial chemoembolization (TACE) with or without prophylactic antibiotic therapy. *Journal of the College of Physicians and Surgeons--Pakistan: JCPSP*.

[30] Serraino C., Elia C., Bracco C. (2018). Characteristics and management of pyogenic liver abscess: a European experience. *Medicine*.

[31] Jiang M., Chen X., Yao H. (2018). The influencing factors for the infection occurring after TACE in patients with liver cancer. *Journal of Interventional Radiology*.

[32] Prajapati H. J., Xing M., Spivey J. R. (2014). Survival, efficacy, and safety of small versus large doxorubicin drug-eluting beads TACE chemoembolization in patients with unresectable HCC. *American Journal of Roentgenology*.

